# Effects of Early Acupuncture Combined with Rehabilitation Training on Limb Function and Nerve Injury Rehabilitation in Elderly Patients with Stroke: Based on a Retrospective Cohort Study

**DOI:** 10.1155/2022/8557936

**Published:** 2022-04-23

**Authors:** Ping Zhang, Guiling Jiang, Qian Wang, Ying Wang, Yihong Ma, Simin Li, Xiubin Li, Hu Li, Xiaomin Xing, Yuzhen Xu

**Affiliations:** ^1^Department of Rehabilitation, The Second Affiliated Hospital of Shandong First Medical University, Taian, 271000, China; ^2^Postdoctoral Workstation, Department of Central Laboratory, The Affiliated Taian City Central Hospital of Qingdao University, Taian, 271000, China; ^3^Department of Neurology, Graduate School of Medical Sciences, Kumamoto University, Kumamoto 860-0811, Japan; ^4^Stomatological Hospital, Southern Medical University, Guangzhou 510515, China; ^5^Department of Neurology, The Second Affiliated Hospital of Shandong First Medical University, Taian, 271000, China

## Abstract

**Objective:**

A case-control study was conducted to explore the effect of acupuncture combined with rehabilitation training on limb function and nerve injury rehabilitation in elderly patients with stroke.

**Methods:**

A total of 72 elderly patients with stroke treated from March 2019 to June 2021 in our hospital were enrolled as the object of study. The clinical data were collected and divided into two groups according to their different treatment methods. The patients cured with routine treatment combined with rehabilitation training were taken as the control group and the patients cured with acupuncture combined with rehabilitation training as the study group. The clinical efficacy was recorded, and the cognition and activities of daily living were evaluated by Terrell Cognitive Assessment scale, limb motor function score, and activities of daily living scale. The National Institutes of Health Stroke Scale (NIHSS) and Glasgow Coma Scale (GCS) were employed to compare the neurological function before and after treatment. Glasgow Outcome Scale (GOS) and Disability Rating Scale (DRS) were adopted to evaluate the functional prognosis. The simplified Fugl-Meyer assessment of motor recovery score was employed to evaluate the limb function of the patients. The Wolf Motor Function Test (WMFT) score was adopted to evaluate the functional rehabilitation effect of the patients. Enzyme-linked immunosorbent assay (ELISA) was adopted to determine the serum neurological function indexes such as nerve growth factor, Smur100B protein, and glial fibrillary acidic protein. The cerebral blood flow (CBF), peak time, average transit time, and cerebral blood volume were measured by CT perfusion imaging, and the incidence of side effects during treatment was recorded.

**Results:**

Regarding the recovery of cognitive function and daily function after treatment, after treatment, the MoCA and ADL scores were increased, and the comparison indicated that the MoCA and ADL scores of the study group were remarkably higher compared to the control group (*P* < 0.05). With regard to the FMA-UE scores after treatment, the Fugl-Meyer scores were gradually increased, and the Fugl-Meyer scores in the study group were remarkably higher compared to the control group (*P* < 0.05) in the next two months. After 2 weeks, 4 weeks, 6 weeks, and 6 weeks of treatment, the WMFT scores gradually increased, and the WMFT score of the study group was remarkably higher compared to the control group. After treatment, the levels of nerve growth factor and S-100B protein were decreased, and the level of glial fibrillary acidic protein was increased. Comparison between the two groups, it indicated the improvement degree of each neurological function index in the study group was remarkably better (*P* < 0.05). With regard to cerebral hemodynamic indexes after treatment, 1 week after treatment, the CBF and average transit time of the observation group were remarkably higher compared to the control group, and the levels of cerebral blood volume and peak time were remarkably lower compared to the control group (*P* < 0.05). After 4 weeks of treatment, the cerebral hemodynamic indexes of the observation group did not change remarkably, and they were all lower than 1 week after the treatment. In the terms of side effects, 1 case of limb dysfunction, 1 case of swallowing dysfunction, 1 case of electrolyte disturbance, and none of infection in the study group, the incidence of adverse reactions was 8.33%. In the control group, there were 3 cases of limb dysfunction, 2 cases of swallowing dysfunction, 2 cases of electrolyte disturbance, and 3 cases of infection, and the incidence of adverse reactions was 27.78%. Compared between groups, the incidence of adverse reactions in the study group was lower (*P* < 0.05).

**Conclusion:**

Early use of acupuncture combined with rehabilitation training has a remarkable therapeutic effect on elderly stroke patients. It can remarkably promote the recovery of the patient's condition, remarkably enhance their neurological function, cognitive function, motor function, and daily life function, and effectively strengthen the patient's prognosis score. It has important clinical application value to reduce the incidence of adverse reactions.

## 1. Introduction

Stroke, also known as “cerebrovascular accident,” is a common neurological disease caused by sudden rupture or obstruction of cerebral blood vessels, with high morbidity and high mortality [1]. With the continuous development of medical diagnosis and treatment, the survival rate of stroke patients increases year by year, but the disability rate remains high, and various functional disorders such as cognition, movement, speech, swallowing, and sensation often occur. It has become the primary cause of disability among adults in China [2, 3]. According to the investigation report [4–6], stroke has the highest incidence, mortality, and disability among all nervous system diseases, and it is the second largest risk factor for death in people over 60 years old. Stroke is the third largest factor affecting human lifespan as a worldwide medical problem. Epidemiological studies have indicated that the incidence of stroke is positively correlated with age.

China is gradually stepping into an aging society, and the incidence of stroke remains high [7]. There are more than 2 million new stroke patients every year. According to statistics, it is found that about 70~80% of patients will have varying degrees of limb dysfunction after stroke, especially upper limb motor dysfunction, which has a high incidence and is difficult to recover, which not only seriously affects the quality of personal daily life but also causes a heavy economic burden to the family and society. Therefore, how to effectively promote the recovery of upper limb motor function in patients with stroke is still a hot and difficult problem in poststroke rehabilitation.

As an important part of traditional Chinese medicine (TCM), acupuncture therapy can treat diseases by stimulating body surface acupoints, reconciling yin and yang, dredging channels and collaterals, and activating blood circulation and qi [8]. At present, it is widely adopted in a variety of nervous system diseases, and it is also one of the traditional rehabilitation treatments. Acupuncture treatment of apoplectic hemiplegia in China has a history of thousands of years, not only has a unique efficacy and advantages but also accumulated a wealth of experience [9]. For example, the argument of “treating impotence and taking Yangming alone” in the Internal Classic of Huangdi emphasizes the treatment of impotence and weakness of the limbs caused by stroke hemiplegia, and the acupoints should be mainly Yangming meridians [10]. The weakness of limbs is mostly caused by deficiency of qi and blood and loss of maintenance of muscles and veins, while Yangming is a meridian with more qi and blood, needling yang can replenish qi and blood, qi and blood are sufficient, muscles and veins are nourished, and the syndrome of impotence should be slow. Acupuncture has unique advantages in the prevention and treatment of stroke, especially when treating hemiplegia, which has definite curative effect, low price, rapid effect, simple, and safe, so it has become an important means of rehabilitation for stroke hemiplegic patients [11].

Modern rehabilitation medicine mainly focuses on rehabilitation training and physiotherapy, which helps to enhance the ability of autonomous movement of the body [12]. Rehabilitation training includes basic training to promote limb movement and coordination and training to promote the recovery of motor function, such as Shaker training, Masako training, and Mendelsohn training [7]. Physiotherapy uses electrical or magnetic stimulation to stimulate nerves and muscles to relieve neuronal palsy. Common treatments include low frequency electrical stimulation, surface myoelectric biofeedback training, and transcranial magnetic stimulation. On the other hand, TCM characteristic rehabilitation attaches importance greatly to when treating stroke sequelae. TCM combined with modern rehabilitation methods when treating stroke sequelae are widely recognized. The Chinese Stroke Rehabilitation Guide points out that TCM has a certain therapeutic effect when treating hemiplegia, dysphagia, and aphasia. Acupuncture is the main method for the treatment of hemiplegia after apoplexy. At present, acupuncture mainly includes head and body acupuncture, neck acupuncture, glossopharyngeal acupuncture, and Xingnao Kaiqiao acupuncture. With the development of medicine, the combination of Chinese and Western therapies and the development of individualized treatment plans are the mainstream direction of rehabilitation in the future.

In recent years, a large number of literatures have reported that acupuncture combined with rehabilitation training is effective when treating motor dysfunction and nerve injury after stroke [13]. However, due to the lack of standardized and unified operation flow between Chinese and western medicine rehabilitation treatment programs, there are many problems such as great differences in intervention measures, nonuniform setting of the control group, and insufficient research sample size. It is still difficult to objectively evaluate the effect of rehabilitation treatment. Currently, some studies have focused on clinical observations of limb function after monotherapy for stroke, and there is a lack of systematic evaluation of the effects of combination therapy. The few studies of combination therapy also have some shortcomings, such as different criteria and poor reliability of control groups. Due to various reasons, acupuncture has not yet established a strict evaluation standard and evaluation system, and the authenticity of its clinical efficacy has not been widely recognized all over the world. The establishment of a system of evaluation that reflects acupuncture therapy consistent with science and widely accepted by the international medical community is a pressing issue at present. The rise and development of evidence-based medicine have had a great impact on the clinical research of acupuncture and moxibustion. Drawing lessons from and applying the evaluation principles of evidence-based medicine has become an important direction of clinical research on acupuncture and moxibustion. Meanwhile, the emergence of evidence-based medicine provides new ideas and theoretical support for the combined research of medical practice from two different medical systems. Based on this, 72 elderly patients with stroke treated from March 2019 to June 2021 in our hospital were studied in this paper, which are reported as follows.

## 2. Patients and Methods

### 2.1. Patient Information

A total of 72 elderly patients with stroke treated from March 2019 to June 2021 in our hospital were enrolled as the object of study, and their clinical data were collected and assigned into two groups according to their different treatment methods. The patients cured with routine treatment combined with rehabilitation training were taken as the control group and the patients cured with acupuncture combined with rehabilitation training as the study group. In the control group, the age ranged from 64 to 85 years old, with an average age of 66.12 ± 6.35 years old, including 20 males and 16 females. In the latter group, the age ranged from 65 to 84 years, with an average age of 67.08 ± 6.79 years, including 19 males and 17 females. The general data of patients were not statistically remarkable. This study was permitted by the medical ethics committee of our hospital, and all patients noticed informed consent.

Selection criteria: (1) referring to the “Key Points for the Diagnosis of Various Major Cerebrovascular Diseases in China 2019” formulated by the Neurology Branch of the Chinese Medical Association, it is in line with the diagnostic points of cerebral infarction and cerebral hemorrhage [13]; (2) brain CT/MRI confirmed the corresponding infarction in the brain, or symptoms and signs lasted for more than 24 hours, or caused death within 24 hours; (3) the onset time of cerebral infarction or cerebral hemorrhage was less than or equal to 90 days; (4) participated in relevant examination and treatment; (5) the clinical data were complete.

Exclusion criteria: (1) complicated with abnormal function of important organs, such as heart, liver, kidney, and lung; (2) mental illness; (3) possible death in the short term; (4) stroke induced by brain tumor, trauma, etc.; (5) complicated by infectious diseases; (6) incomplete clinical data.

### 2.2. Treatment Methods

The control group was given conventional treatment combined with rehabilitation training: (1) conventional treatment, 100 mg of aspirin each time, once a day; 75 mg of clopidogrel hydrogen sulfate tablets each time, once a day; conventional hypolipidemic, hypoglycemic, and hypotensive; (2) rehabilitation training, motor function training, 30 minutes per training, exercise 1-2 times a day; language training, cognitive function training, 30 minutes per training, 1 training per day; daily life ability training, 30 minutes per training, every day 1 training session.

The study group received acupuncture treatment on the basis of the control group: meridian acupuncture to refresh the mind, dredge the meridians, and reconcile yin and yang. The main acupoints were Fenglong, Yongquan, Zusanli, Yanglingquan, Shuigou and Weizhong, Quchi point, Hegu point, Sanyinjiao point, Neiguan point, Baihui point, and Chize point. Addition and subtraction according to the symptoms: the mouth and eyes are skewed, the eyes cannot be closed, Jiajiache point, Dicang point, Chengli point, Yingxiang point; lower limb dysfunction plus ring jumping blood, and Taichong acupoint; upper limb dysfunction plus Waiguan acupoint, Shou Sanli acupoint, shoulder Kuang acupoint, shoulder Zhen acupoint, and shoulder well acupoint; speech unfavorable plus Tongli acupoint, Yuye acupoint, Lianquan acupoint, and Jinjin acupoint. Supine position, acupoint skin disinfection, Sanyinjiao acupoint tonifying method, Neiguan acupoint diarrhea method, Shuigou acupoint Finch cough method, straight needling at Shize acupoint and Weizhong acupoint, and lifting and insertion method to make the limbs have a sense of twitching and numbness. The rest of the acupoints was cured with the method of deficiency, replenishment, and catharsis; and the bilateral acupoints were cured with acupuncture on the affected side. About 25 min was retained after acupuncture at the affected side, and acupuncture was performed once at intervals of 5 min. Both groups were treated continuously for 8 weeks.

### 2.3. Observation Index

#### 2.3.1. Evaluation Standard of Curative Effect

After 8 weeks of treatment, the clinical effects were evaluated. The cure indicated that the neurological function of the patient recovered completely, the clinical symptoms basically disappeared or disappeared completely, and CT examination indicated that the focus recovered completely and could live a normal life; for improvement, the neurological function of the patient partially returned to normal, the clinical symptoms enhanced, CT examination indicated that there were still intracranial lesions or lesions were enlarged, and daily life could basically take care of themselves. Ineffective for patients with no change in neurological function or even aggravated, there are serious mental or motor disorders, CT examination of patients with intracranial degenerative lesions, and life is still unable to take care of themselves. Clinical effective rate = (cure + improvement) cases/total cases × 100%.

#### 2.3.2. Evaluation of the Degree of Neurological Impairment

The neurological function of the two groups was recorded before and 8 weeks after treatment, and the neurological deficit was scored with the NIHSS [14]. The scale included 12 items, such as level of consciousness, gaze, visual field, upper limb movement, lower limb movement, ataxia, facial paralysis, sensation, language, dysarthria, neglect, and distal motor function.

#### 2.3.3. Coma Degree Assessment

GCS was used to evaluate the coma degree of the patients, including eye opening, language, and exercise, with a full score of 15 [15]. The lower the score, the more serious the coma.

#### 2.3.4. Functional Prognosis Assessment

GOS was adopted to grade the degree of disability of the patients, which was assigned into death (grade I), vegetative state (grade II: long-term coma, eye opening, periodic eye opening-awake), severe disability (grade III unable to take care of themselves, with severe mental and physical disabilities, conscious), moderate disability (grade IV: able to take care of themselves in daily life, and able to engage in some daily activities in specialized environments), work or activities, and good recovery (grade V: return to normal life, self-care, but there may be minor neurological or pathological defects) 5 grades [16].

#### 2.3.5. Cognitive Function Assessment

Cognitive function recovery was assessed using the Montreal Cognitive Assessment (MoCA), with 11 items, each with a score of 0-30, with higher scores indicating better cognitive function [17].

#### 2.3.6. Motor Function Evaluation

The recovery of motor function was assessed using the Fugl-Meyer score [18], with a score ranging from 0-100, with higher scores indicating better motor function.

#### 2.3.7. Living Ability Assessment

The recovery of living ability was assessed by the activity of daily living scale (ADL), with a score of 0-100 [19]. The higher the score, the better the daily living ability of the patient, and a score of 61 or more indicated a good prognosis.

#### 2.3.8. Upper Limb Functional Training Effect Score

The upper limb functional training of patients was evaluated by the WMFT with a total of 15 items, all of which were scored using a 6-level scoring method [20]. The higher the score, the better the functional training effect of the patients.

#### 2.3.9. Neurological Rehabilitation Index

The serum neurological function indexes such as nerve growth factor, Smur100B protein, and glial fibrillary acidic protein were measured by enzyme-linked immunosorbent assay (ELISA), and the levels of amino acid neurotransmitters such as glutamic acid, *γ*-aminobutyric acid, aspartic acid, and glycine were measured by liquid phase mass spectrometry. Cerebral blood flow, time to peak, mean transit time, and cerebral blood volume were measured by CT perfusion imaging.

### 2.4. Statistical Analysis

SPSS 22.0 statistical software was employed for statistical analysis of data, measurement data were presented as mean ± standard deviation, and *t* test was adopted; count data was presented as %, and *χ*^2^ test was adopted. *P* < 0.05 was considered remarkable difference.

## 3. Results

### 3.1. Comparison of Therapeutic Effects

First of all, we compared the therapeutic effects. In the study group, 23 cases were cured, 10 cases improved, 3 cases ineffective, no cases poor, and the effective rate was 91.67%. In the control group, 17 cases were cured, 9 cases improved, and 10 cases ineffective. The effective rate was 72.22%. The effective rate of the study group was higher compared to the control group (*P* < 0.05). All the results are indicated in Figure 1.

### 3.2. Two Groups of Patients NIHSS, GCS, and DRS Score Comparison

We compared the NIHSS, GCS, and DRS scores. Before treatment, there exhibited no remarkable difference (*P* > 0.05). After treatment, the NIHSS, GCS, and DRS scores of patients were decreased. Compared between the two groups, the NIHSS, GCS, and DRS scores of the study group were remarkably lower (*P* < 0.05). All results are indicated in Table 1.

### 3.3. Comparison of Cognitive Function and Daily Function Recovery of Patients after Treatment

We compared the recovery of cognitive function and daily function after treatment. Before treatment, there exhibited no remarkable difference (*P* > 0.05). After treatment, the MoCA score and ADL score were increased. Compared with the two groups, the MoCA score and ADL score of the study group were remarkably higher (*P* < 0.05). All results are indicated in Table 2.

### 3.4. Fugl-Meyer Scores Comparison

We compared the FMA-UE scores after treatment. Before treatment, there exhibited no remarkable difference in Fugl-Meyer scores (*P* > 0.05). After 2 weeks, 4 weeks, 6 weeks, and 6 weeks of treatment, the Fugl-Meyer scores were gradually increased, and the Fugl-Meyer scores in the study group were remarkably higher compared to the control group (*P* < 0.05). The specific results are indicated in Table 3.

### 3.5. Comparison of Neurological Function Indexes before and after Treatment

We compared the neurological function indexes before and after treatment. Before treatment, there exhibited no remarkable difference in the neurological function indexes (*P* > 0.05). After treatment, the levels of nerve growth factor and S-100B protein were reduced, and the level of glial fibrillary acidic protein was increased. Compared with the two groups, the improvement of various neurological function indexes in the study group was remarkably better (*P* < 0.05). All results are indicated in Table 4.

### 3.6. Comparison of Cerebral Hemodynamic Indexes after Treatment

We compared the cerebral hemodynamic indexes of patients after treatment. One week after treatment, the CBF and average transit time of the observation group were remarkably higher compared to the control group, and the levels of cerebral blood volume and peak time were remarkably lower compared to the control group (*P* < 0.05). After 4 weeks of treatment, the cerebral hemodynamic indexes of the observation group did not change remarkably, and the cerebral hemodynamic indexes of the control group were all lower than 1 week after the treatment. All results are indicated in Table 5.

### 3.7. Comparison of Adverse Reactions

We compared the adverse reactions. In the research group, there was 1 case of limb dysfunction, 1 case of swallowing dysfunction, 1 case of electrolyte disturbance, and none of infection. The incidence of adverse reactions was 8.33%. In the control group, there were 3 cases of limb dysfunction, 2 cases of swallowing dysfunction, 2 cases of electrolyte disturbance, and 3 cases of infection, and the incidence of adverse reactions was 27.78%. Compared between groups, the incidence of side effects in the study group was lower (*P* < 0.05). All results are indicated in Figure 2.

## 4. Discussion

Stroke includes ischemic stroke and hemorrhagic stroke and is a kind of disease caused by cerebral vascular obstruction or hemorrhage and interruption of cerebral vascular blood flow, which has the characteristics of high incidence, high mortality, high disability rate, high recurrence rate, and high medical cost [20]. The China Stroke Prevention and Treatment Report 2019 points out that stroke has become the leading cause of death among Chinese residents due to disease [21]. In 2017, the prevalence rate of ischemic stroke in China accounted for 82.4% of stroke, and the stroke mortality rate increased to 149/100000. The recurrence rate of stroke within 3 months indicated a downward trend, in which the recurrence rate of hemorrhagic stroke within 3 months was much lower compared to ischemic stroke. After stroke, 70~80% of patients will have motor dysfunction and a serious decline in physical activity and activities of daily living, which not only brings great pressure on the patient's body and mind but also increases the burden on the patient's family.

At present, many scholars have explored the correlation between these factors and limb dysfunction after stroke from the aspects of sex, age, location of the disease, marital status, depression, treatment methods, treatment intervention time, and the degree of neurological impairment at admission [22]. Most scholars believe that the degree of limb dysfunction after stroke is related to age, marital status, depression, rehabilitation training, treatment and intervention time after onset, and the degree of neurological impairment. A survey of 705 stroke inpatients in Daqing found that 64% of stroke patients had limb dysfunction [22]. Among them, advanced age, no spouse, hypertension, heart disease, severe neurological impairment on admission, and depression are the risk factors of limb dysfunction after stroke. Regular exercise, high subjective support, and high utilization of support can reduce the risk of motor dysfunction after stroke [23]. A retrospective study of 210 stroke patients with different course of stroke pointed out that the distribution of disability in patients with limb dysfunction with a course of 6, 12, and 18 months was mostly concentrated in moderate and severe disabilities. And the proportion of moderate and severe disability in patients with different course of disease is similar, and this study suggests that the recovery of limb function of stroke patients is slow after 6 months. Some scholars also believe that early intervention can more effectively promote the recovery of limb function after stroke.

Some scholars have long discussed the effect of standardized tertiary rehabilitation on the improvement of patients with limb dysfunction, including physiotherapy and occupational therapy [24]. Studies have also confirmed the promoting effect of standardized rehabilitation on the improvement of limb function. For stroke patients with unfavorable limb movement, in addition to routine limb function training, transcranial magnetic stimulation, and some other exercise therapies are often adopted to promote the recovery of their function. The study found that repetitive transcranial magnetic stimulation can effectively relieve the spasticity of the limbs in patients with stroke and reduce the degree of neurological deficits. The earlier the intervention, the better the effect. The study by Wang and others found that the mirror therapy combined with the conventional rehabilitation training group enhanced the upper limb motor function, daily living ability, and electromyographic signal of stroke patients better than the conventional rehabilitation training group [25]. Therapy is more conducive to the recovery of patients' limb function and helps patients regain their independent living ability. Han et al.'s research found that mirror therapy combined with suspension training could also strengthen the limb balance ability of stroke patients [26]. In addition, rope therapy, ultrasonic electrical stimulation, and PNF technology have all been confirmed to enhance the therapeutic effect of conventional rehabilitation therapy and have a positive effect on the gait and balance of poststroke hemiplegia patients.

In TCM, the sequelae of stroke belong to the category of “partial withering” and “partial abandonment” [27]. The pathological basis is qi and blood deficiency and vein stasis. Acupuncture can ensure adequate blood perfusion of brain tissue and prolong the tolerance time of the body to cerebral ischemia; acupuncture can also stimulate vascular self-regulation, relieve constriction of cerebral vessels, and enhance microcirculation; acupuncture can promote the recovery of nerve function, which is conducive to rehabilitation; acupuncture can dilate the blood vessels of the brain and limbs, facilitate the establishment of cerebral vascular collateral circulation, and promote the functional recovery of motor neurons [27]. Many studies have confirmed the effectiveness of acupuncture when treating hemiplegic patients, and acupuncture is also recommended in Chinese guidelines for the treatment of limb dysfunction after cerebral infarction (grade I recommendation, level A evidence). According to the existing literature, acupuncture can affect the signal pathways of Notch, PDGF-*β*, and VEGF; promote the formation of micro vessels; reduce the occurrence of inflammatory reaction; slow down the apoptosis of neurons; and effectively control the focus area.

A real-world study on the efficacy of acupuncture when treating stroke found that on the basis of conventional rehabilitation therapy, adding acupuncture can effectively improve the MBI score and reduce the MRS score of patients [27]. The patients' recovery of limb function was accelerated. In addition, for patients with hemiplegia after cerebral infarction, FMA scores were higher with electroacupuncture combined with moxibustion after 3 months of treatment. There exhibited no remarkable difference in curative effect between the combined moxibustion groups. Electroacupuncture combined with moxibustion was superior to acupuncture alone in improving limb function. A real-world clinical study of 302 stroke patients conducted by Huang et al. found that the BI scale score of the acupuncture group at 3 months was higher compared to the conventional drug treatment group, and the MRS scale score was lower compared to the conventional drug treatment group [28]. In the real world, acupuncture treatment enhances function of stroke patients better than conventional drug treatment. The study by Liu and others found that for patients with flaccid paralysis, the combination of the major meridian method combined with staged acupuncture has a more remarkable effect and effectively enhanced the patient's FMA score and daily living ability [29]. Song and others pointed out that, whether it is cerebral infarction or cerebral hemorrhage, the combined therapy of scalp acupuncture and body acupuncture combined with Bobath therapy can improve their neurological deficit and limb mobility and relieve muscle spasm [30]. Yang and others conducted a systematic review of 9 randomized and quasirandomized clinical trials and the treatment of a total of 931 patients with cerebral infarction and found that in reducing the disability rate of patients with cerebral infarction, Xingnao Kaiqiao acupuncture therapy was remarkably better [31]. In the drug and conventional acupuncture groups, the long-term efficacy of Xingnao Kaiqiao acupuncture therapy was also remarkable. Wu and other scholars performed comprehensive surface electromyography acupuncture treatment on 80 patients with poststroke lower limb spasm. Before acupuncture, the surface electromyography of the affected limb was measured, and the diseased muscle was accurately located before acupoint selection. This method can effectively relieve the pain. The patient's lower extremity spasticity was improved, and the motor function recovery of the lower extremity was promoted. Some scholars have studied meridian acupuncture and acupuncture points and found that the combination of the above acupuncture methods in conventional rehabilitation therapy could improve the motor function of stroke patients.

This study showed that early use of acupuncture combined with rehabilitation training could remarkably promote the neurological damage and enhance the recovery of neurological function in elderly stroke patients. After the central nervous system was damaged, part or all of its function could be restored through rehabilitation therapy. Early rehabilitation training can activate the damaged nerve tissue by the axons of healthy nerve tissue, thereby regenerating and restoring brain function. Early rehabilitation training after treatment for stroke patients is beneficial to limb blood circulation, effectively preventing muscle atrophy and enhancing neurotrophic function. In this study, from the perspective of mental recovery, the NIHSS scores of the patients in the study group cured with acupuncture combined with rehabilitation training were remarkably lower compared to the control group with only limb rehabilitation training. For the patients with only limb rehabilitation training, it suggests that acupuncture combined with rehabilitation training can remarkably promote cognition, limb function, and daily living ability of stroke patients, and regardless of the prognosis or the results of self-assessment of life quality after treatment, the therapeutic effect of acupuncture combined with rehabilitation training better. Among the enrolled acupoints in this study, acupuncture at Yongquan and Sanyinjiao can nourish yin and tonify kidney; acupuncture at Baihui and Zusanli can regulate spleen and stomach, dredge channels, and collaterals and enhance blood circulation in the brain; Weizhong, Shusanli, Fenglong, Taichong, Shize, Huantiao, Quchi, Waiguan, Neiguan, and shoulder Zhen acupuncture can promote blood circulation, disperse blood stasis, relax muscles, and dredge collaterals, which is conducive to the recovery of normal function of the upper and lower limbs. Acupuncture at Yuye acupoint, Jinjin acupoint and Lianquan acupoint can promote the recovery of language function; acupuncture at cheek car acupoint, Dicang acupoint and Yingxiang acupoint can correct mouth and eye deviation; acupuncture at Shenjue acupoint and Baihui acupoint can promote local blood circulation and increase CBF. It is beneficial to the functional recovery of nerve cells.

Nerve growth factor, glial fibrillary acidic protein, and Smur100B protein are all indicators of neurological function, and their changes are closely related to GCS score. In this study, the improvement of neurological function indexes in the study group was remarkably higher compared to the control group, suggesting that the combination of acupuncture and rehabilitation training is more beneficial to the recovery of neurological function of patients. It is proved that acupuncture and rehabilitation training are feasible from the micro level. Some studies have indicated that hyperbaric oxygen adjuvant therapy can enhance the stress state of patients and promote the supply of blood oxygen. Other studies have pointed out that acupuncture combined with rehabilitation training can increase the arterial blood flow velocity, enhance the cerebral arterial blood flow capacity, and effectively strengthen the circulatory metabolic system. In this study, the hemodynamic indexes of patients in the observation group were more stable after operation. The prognosis of the patients in the study group indicated that the GOS score was higher, and the incidence of side effects was lower, indicating that the functional prognosis of the patients in the observation group was better.

Conclusively, the clinical effect of rehabilitation training combined with acupuncture when treating elderly patients with stroke is remarkable, which can remarkably enhance the limb function and activities of daily life of the patients and promote the rehabilitation of their nerve injury. The combination scheme has a certain prospect of rehabilitation application and promotion.

## Figures and Tables

**Figure 1:** Comparison of therapeutic effects between the two groups.

**Figure 2:** Comparison of adverse reactions between the two groups.

**Table 1:** Two groups of patients NIHSS, GCS, and DRS score comparison ($\bar{x}\pm s$, points).

Group	*N*	NIHSS score		GCS score		DRS score	
		Before treatment	After treatment	Before treatment	After treatment	Before treatment	After treatment
C group	36	30.63 ± 3.46	21.33 ± 3.42^a^	5.36 ± 1.23	9.44 ± 2.48^a^	21.77 ± 3.38	17.48 ± 2.45^a^
R group	36	30.82 ± 3.35	15.36 ± 2.28^b^	5.74 ± 1.46	12.38 ± 3.41^b^	21.56 ± 3.34	11.34 ± 2.16^b^
*t*		0.237	8.715	1.194	4.184	0.265	11.279
*P*		>0.05	<0.01	>0.05	<0.01	>0.05	<0.01

Note: comparison before and after treatment in the control group, ^a^*P* < 0.05; comparison of the research group before and after treatment, ^b^*P* < 0.05.

**Table 2:** Comparison of cognitive, physical function and daily function recovery of patients after treatment ($\bar{x}\pm s$, points).

Group	*N*	NIHSS score		GCS score	
		Before treatment	After treatment	Before treatment	After treatment
C group	36	14.23 ± 1.87	20.17 ± 3.36	65.36 ± 1.23	75.56 ± 9.41
R group	36	14.78 ± 1.26	25.28 ± 3.95	65.74 ± 1.46	88.42 ± 10.86
*t*		1.463	5.912	1.194	5.370
*P*		>0.05	<0.01	>0.05	<0.01

**Table 3:** Comparison of Fugl-Meyer scores between the two groups before and after intervention ($\bar{x}\pm s$, points).

Group	*N*	Before treatment	After 2 weeks of treatment	After 4 weeks of treatment	After 6 weeks of treatment	After 8 weeks of treatment
C group	36	33.54 ± 7.06	39.03 ± 6.89^a^	44.25 ± 7.58^a^	46.08 ± 8.13^a^	49.17 ± 9.01^ba^
R group	36	32.98 ± 6.21	45.79 ± 7.03^ab^	52.38 ± 8.27^ab^	55.43 ± 9.18^ab^	59.37 ± 10.38^ab^
*t*		0.357	4.121	4.348	4.575	4.453
*P*		>0.05	<0.01	<0.01	<0.01	<0.01

Note: compared with the control group, ^a^*P* < 0.05; compared with this group before treatment, ^b^*P* < 0.05.

**Table 4:** Comparison of neurological function indexes in two groups of patients before and after treatment ($\bar{x}\pm s$).

Group		*N*	Nerve growth factor (ng/L)		Glial fibrillary acidic protein (ng/L)		S-100B egg white (*μ*g/L)	
			Before treatment	After treatment	Before treatment	After treatment	Before treatment	After treatment
C group	36	0.71 ± 0.15	1.66 ± 0.28^a^	5.58 ± 0.93	1.19 ± 0.25^a^	0.48 ± 0.05	0.23 ± 0.02^a^	
R group	36	0.72 ± 0.11	2.14 ± 0.26^b^	5.56 ± 1.04	0.63 ± 0.11^b^	0.46 ± 0.06	0.12 ± 0.04^b^	
*t*		0.323	7.537	1.376	12.302	1.536	14.758	
*P*		>0.05	<0.01	>0.05	<0.01	>0.05	<0.01	

Note: comparison of control group before and after treatment, ^a^*P* < 0.05; comparison of the research group before and after treatment, ^b^*P* < 0.05.

**Table 5:** Comparison of cerebral hemodynamic indexes between the two groups of patients after treatment ($\bar{x}\pm s$).

Group	*N*	CBF (ml/(100 g·min))		Cerebral blood volume (s)		Peak time (s)		Passing time (ml/100 g)	
		1 week after treatment	4 weeks after treatment	1 week after treatment	4 weeks after treatment	1 week after treatment	4 weeks after treatment	1 week after treatment	4 weeks after treatment
C group	36	28.66 ± 5.61	23.08 ± 4.15	19.06 ± 2.33	20.05 ± 2.16	2.93 ± 0.34	3.46 ± 0.51	1.53 ± 0.23	1.14 ± 0.16
R group	36	34.31 ± 6.34	33.54 ± 6.26	16.51 ± 1.89	15.91 ± 1.74	2.03 ± 0.25	2.11 ± 0.34	2.26 ± 0.47	2.28 ± 0.41
*t*		4.004	8.356	5.100	8.956	12.796	13.215	8.371	15.541
*P*		<0.01	<0.01	<0.01	<0.01	<0.01	<0.01	<0.01	<0.01

Note: comparison before and after treatment in the control group, ^a^*P* < 0.05; comparison of the research group before and after treatment, ^b^*P* < 0.05.

## Data Availability

The study data presented may be made available from the corresponding author upon reasonable request.

## References

[1] Xu Y., Wang Q., Chen J., Ma Y., Liu X. (2020). Updating a strategy for histone deacetylases and its inhibitors in the potential treatment of cerebral ischemic stroke. *Disease Markers*.

[2] Wang J., Hu Z., Yang S. (2018). Inflammatory cytokines and cells are potential markers for patients with cerebral apoplexy in intensive care unit. *Experimental and Therapeutic Medicine*.

[3] Xu Y., Wang K., Wang Q., Ma Y., Liu X. (2021). The antioxidant enzyme PON1: a potential prognostic predictor of acute ischemic stroke. *Oxidative Medicine and Cellular Longevity*.

[4] Wang Q., Wang K., Ma Y., Li S., Xu Y. (2021). Serum galectin-3 as a potential predictive biomarker is associated with poststroke cognitive impairment. *Oxidative Medicine and Cellular Longevity*.

[5] Chen J., Li S. (2019). Clinical study of neurology nursing on cerebral apoplexy rehabilitation. *Translational Neuroscience*.

[6] Wang X., Wang Q., Wang K. (2022). Is immune suppression involved in the ischemic stroke? A study based on computational biology. *Frontiers in Aging Neuroscience*.

[7] Yan B., Zhang H., Liu J. (2021). Application of quantitative CT imaging in rehabilitation nursing of cerebral apoplexy patients. *Pakistan Journal of Medical Sciences*.

[8] Pokhrel B., Khanal S., Chapagain P., Sedain G. (2021). Pituitary apoplexy complicated by cerebral infarction: a case report. *Journal of the Nepal Medical Association*.

[9] Jing T. (2021). Observation on the efficacy of Tongnao Huoluo acupuncture therapy combined with Buyang Huanwu decoction when treating stroke. *Inner Mongolia TCM*.

[10] Feng Q., Lina L. (2021). Effect of acupuncture combined with soothing the liver and relieving depression on cognitive impairment after stroke of liver-qi stagnation and its effect on the level of neurotransmitters. *Clinical medical research and practice*.

[11] Luo M., Duan Z., Song X. (2022). Effects of optimized acupuncture and moxibustion treatment on depressive symptoms and executive functions in patients with post-stroke depression: study protocol for a randomized controlled trial. *Frontiers in Neurology*.

[12] Yangyang S., Li Chaosheng L., Jianfang L. (2022). Analysis of the effect of task-oriented training combined with rehabilitation training on dysphagia after stroke. *Medical higher Vocational Education and Modern Nursing*.

[13] Xu J. J., Song Y., Jiang P. (2019). Effect of prior stroke on long-term outcomes of percutaneous coronary interventions in Chinese patients: A large single-center study. *Catheterization and Cardiovascular Interventions*.

[14] Chalos V., van der Ende N. A. M., Lingsma H. F. (2020). National Institutes of Health Stroke Scale: an alternative primary outcome measure for trials of acute treatment for ischemic stroke. *Stroke*.

[15] Estévez-Báez M., Machado C., García-Sánchez B. (2019). Autonomic impairment of patients in coma with different Glasgow coma score assessed with heart rate variability. *Brain Injury*.

[16] Mohamed F. F., Ayman M. I., Amer M. (2021). Decompressive craniectomy in patients with malignant middle cerebral artery infarction: prognostic factors and timing dilemma. *The Medical Journal of Cairo University*.

[17] Smith T., Gildeh N., Holmes C. (2007). The Montreal Cognitive Assessment: validity and utility in a memory clinic setting. *The Canadian Journal of Psychiatry*.

[18] Rech K. D., Salazar A. P., Marchese R. R., Schifino G., Cimolin V., Pagnussat A. S. (2020). Fugl-Meyer assessment scores are related with kinematic measures in people with chronic hemiparesis after stroke. *Journal of Stroke and Cerebrovascular Diseases*.

[19] Jin T., Lian W., Xu K. (2021). Effect of combination invasive intracranial pressure (ICP) monitoring and transcranial Doppler in the treatment of severe craniocerebral injury patients with decompressive craniectomy. *Ann. Palliat. Med*.

[20] Zhang M., Chen J., Ling Z. (2022). Quantitative evaluation system of upper limb motor function of stroke patients based on desktop rehabilitation robot. *Sensors*.

[21] Tao P., Ji J., Gu S., Wang Q., Xu Y. (2022). Progress in the mechanism of autophagy and traditional Chinese medicine herb involved in dementia. *Frontiers in Pharmacology*.

[22] Juan L., Yumei L., Yuqiu Z., Yingli L., Wei Y. (2017). Study on disability status and influencing factors of stroke patients in Daqing City. *China Journal of Rehabilitation Medicine*.

[23] Weixia S., Yumei L., Yujing S., Lina M., Li L. (2020). Analysis of the level of social participation and influencing factors of disabled patients after stroke with different course. *China Nursing Management*.

[24] Tan Z., Xiaoli F., Yu W., Zhongzhong X. (2019). Relationship between H-type hypertension and acute cerebral infarction Oxfordshire Community Stroke Project classification and short-term prognosis. *Chinese General Medicine*.

[25] Zhuang J. Y., Ding L., Shu B. B., Chen D., Jia J. (2021). Associated mirror therapy enhances motor recovery of the upper extremity and daily function after stroke: a randomized control study. *Neural Plasticity*.

[26] Rong H., Wenguang X., Yangpu Z., Chanjuan Z. (2021). Rehabilitation effect of suspension training combined with mirror therapy on balance function of lower limbs in patients with cerebral infarction. *Nerve Injury and Function Reconstruction*.

[27] Yunxia H. (2020). *Comparative Benefit Study Analyzed the Maximum Benefit Scheme of Acupuncture when Treating Motor Dysfunction after Stroke*.

[28] Zhan J., Xiong B., Zhang P. (2021). Abdominal acupuncture as an adjunctive therapy for the recovery of motor function after stroke: a systematic review and meta-analysis of randomized controlled trials. *Frontiers in Neurology*.

[29] Zhang Z. Q., Li K. P., He J. (2020). Acupuncture of fascia points to relieve hand spasm after stroke: a study protocol for a multicenter randomized controlled trial. *Trials*.

[30] Jinli Z., Jinbo C., Pingxuan W. (2020). Application of acupuncture combined with exercise therapy in promoting the rehabilitation of stroke patients with hemiplegia. *Clinical Research in Traditional Chinese Medicine*.

[31] Yang Z. X., Xie J. H., Liu Y. P. (2015). Systematic review of long-term Xingnao Kaiqiao needling effcacy in ischemic stroke treatment. *Neural Regeneration Research*.

